# Weak Signal Enhance Based on the Neural Network Assisted Empirical Mode Decomposition

**DOI:** 10.3390/s20123373

**Published:** 2020-06-15

**Authors:** Kai Chen, Kai Xie, Chang Wen, Xin-Gong Tang

**Affiliations:** 1 National Demonstration Center for Experimental Electrical & Electronic Education, Yangtze University, Jingzhou 434023, China; 201703455@yangtzeu.edu.cn; 2 School of Computer Science, Yangtze University, Jingzhou 434023, China; 400100@yangtzeu.edu.cn; 3 School of Electronic and Information, Yangtze University, Jingzhou 434023, China; 4 Key Laboratory of Exploration Technologies for Oil and Gas Resources (Yangtze University), Ministry of Education, Wuhan 430100, China; tangxg@yangtzeu.edu.cn

**Keywords:** weak signal, strong background noises, complete ensemble empirical mode, graphical processing unit, parallel computing, cyclic neural network, generative adversarial network

## Abstract

In order to enhance weak signals in strong noise background, a weak signal enhancement method based on EMDNN (neural network-assisted empirical mode decomposition) is proposed. This method combines CEEMD (complementary ensemble empirical mode decomposition), GAN (generative adversarial networks) and LSTM (long short-term memory), it enhances the efficiency of selecting effective natural mode components in empirical mode decomposition, thus the SNR (signal-noise ratio) is improved. It can also reconstruct and enhance weak signals. The experimental results show that the SNR of this method is improved from 4.1 to 6.2, and the weak signal is clearly recovered.

## 1. Introduction

Traditional signal analysis and processing starts from the theory of Fourier analysis. However, Fourier analysis is only applicable to the global transformation of stationary and linear signals. Therefore, it is impossible to describe the time-frequency local characteristics of signals. Especially in the case of strong noise, the traditional Fourier transform is difficult to deal with the weak signal in the background of strong noise under the premise of ensuring high fidelity. Recently, some scholars have proposed a non-linear method of wavelet threshold [1,2], but the wavelet basis function is fixed, thus it cannot match all real signals. To be precise, wavelet analysis does not have the characteristics of self-adaptation. Once a wavelet basis function is selected, it will be used to analyze all data, if the selected wavelet decomposition is inappropriate, it will limit its denoising effect. Thus, it is very difficult to enhance the weak signal in a low SNR environment [3,4,5]. In 1998, Huang proposed a Hilbert–Huang transform (HHT) [6] signal processing method based on the Hilbert transform (Hilbert–Huang transform is based on two parts. The first part is empirical mode decomposition, and the second part is Hilbert spectrum analysis) This method has improved the processing of non-linear and non-stationary signals [7,8]. The key part of the HHT method is the EMD (empirical mode decomposition), which decomposes the signal into a series of sub-signals called IMFs (intrinsic mode functions). It can separate the intrinsic modal component from the pseudo component or the noise concentration, but it cannot select the IMF adaptively and enhance the weak signal adaptively, thus it is easy to cause modal anomalies, but the Hilbert–Huang transformation is an empirical approach with many deficiencies [9,10], such as mode mixing, boundary effects, and instantaneous frequency errors, etc. In order to resolve these defects, our paper proposes a method of fast enhancement of weak signals based on the optimized EMD and neural network (EMDNN) model. The EMDNN method can adaptively select effective intrinsic [11] modal components and adaptively enhance instantaneous amplitude to reconstruct weak signals. With the increasing pace of people’s exploration of the objective world, the 3D seismic exploration technology is also gradually in-depth, but if the SNR of 3D seismic signal is low, it will affect the follow-up signal processing and interpretation work, which may lead to a large miscalculation. Therefore, it is of practical significance to study efficient 3D seismic signal denoising algorithm [12].

## 2. Weak Signal Reconstruction Method under EMDNN Model

This paper presents the EMDNN model, which is mainly used to detect and reconstruct the weak signals in strong noise background, and reduce the problem of mode mixing [13,14] (when the signal is screened, some IMF components with different time scales will appear, which is called mode mixing). This method decomposes the modal function from high-frequency to low-frequency distribution [15], thereby reducing the loss of effective information. By applying this method to weak signal processing and reconstruction, we cannot only get rid of the constraints of weak signal linearity and stationarity but also achieve good accuracy in both time and frequency [16]. At the same time, it also has complete self-adaptiveness, and on the basis of suppressing all kinds of strong and weak noises, effective signals are highlighted to improve the accuracy of reconstructed signals. In addition, LSTM (long short-term memory) [17], GAN (generative adversarial networks) [18,19] are used to assist this method, which further improves the recovery and enhancement of weak signals.

The weak signal data and the processing flow of the algorithm bring great challenges in the weak signal enhancement method proposed in our paper. In this section, the first step is to pre-process the original weak signal. The second step is to use the complementary set empirical mode decomposition method to decompose the pre-processed signal and obtain the intrinsic modal component. In the third step, the LSTM model is trained by correlation computation to select the effective intrinsic modal components adaptively, and the instantaneous amplitude and phase of the instantaneous frequency are obtained by the Hilbert transform. In the fourth step, we reconstruct the instantaneous phase and amplitude to recover the weak signal without enhancement. Finally, the GAN model was trained to generate enhanced weak high-definition signals. Figure 1 shows the flow chart of our method. We used the three-dimensional seismic data [20] as the input signal. The three-dimensional seismic signal is the three-dimensional spatial data obtained from the propagation route and time of the artificially excited seismic wave in the underground strata [21,22].

### 2.1. Original Signal Pre-Processing

We first pre-process the input signal. In order to prevent the common denoising method from destroying the smoothness and continuity of the horizontal slice of the seismic signal, we use non-linear wavelet transform threshold value method to denoise the seismic signal to eliminate the regular noise in the original signal [23].

### 2.2. Empirical Mode Decomposition

After we get the one-dimensional signal after pre-processing, we start empirical mode decomposition. Adding different amplitudes of Gaussian white noise *λ*_0_*w*(*i*) to the original signal *x* (*λ*_0_ is the amplitude, *w*(*i*) is the white noise that achieves a zero average unit variance), *x*(*i*) = *x* + *λ*_0_*w*(*i*), *I* = 1, 2, 3, …, n or the actual data is subjected to the empirical mode decomposition (EMD), The integral set components of the first intrinsic mode function EMD are obtained by averaging the components of the first intrinsic mode function (IMF) *d*_1_(*i*):

(1) $${\tilde{s}}_{1}=\frac{1}{n}\sum_{i=1}^{n}d_{1}\left(i\right)={\bar{s}}_{1}$$

Let *E_j_* (*) is the operator of the *j*-th mode generated after EMD decomposition, and the first remaining component can be calculated from the first step *r*_1_:

(2) $$r_{1}=x-{\tilde{s}}_{1}$$

The first mode component is obtained by EMD decomposition: *r*_1_ + *λ*_1_*E*_1_[*w*(*i*)], *I =* 1, 2, 3, …, *n*; The EMD decomposition is performed again, and the available intrinsic mode components obtained after decomposition are summed and averaged to obtain the second set of EMD intrinsic mode functions:

(3) $${\tilde{s}}_{2}=\frac{1}{n}\sum_{i=1}^{n}E_{1}\left\{r_{1}+\lambda_{1}E_{1}\left[w\left(i\right)\right]\right\}$$

And the *k*-th residual component can be obtained through loop iteration *r_k_*:

(4) $$r_{k}=r_{\left(k-1\right)}-{\tilde{s}}_{k}$$

And the complete set component of the (*k* + 1)-th EMD is obtained from the intrinsic mode component formula obtained through EMD decomposition:

(5) $${\tilde{s}}_{\left(k+1\right)}=\frac{1}{n}\sum_{i=1}^{n}E_{1}\left\{r_{k}+\lambda_{k}E_{k}\left[w\left(i\right)\right]\right\}$$

Repeated iteration calculations to the remaining components cannot be performed in the EMD decomposition, the remaining components satisfy the IMF condition. After satisfying the condition after the *m*-th iteration, the original signal is subtracted from the sum of the intrinsic modal functions obtained by the decomposition to obtain the final residual component *r_m_*:

(6) $$r_{m}=x-\sum_{j=1}^{m}{\tilde{s}}_{j}$$

Thus, the original signal can be reconstructed:

(7) $$x=\sum_{j=1}^{m}{\tilde{s}}_{j}+r_{m}$$

### 2.3. Adaptive Selection of Effective Inherent Modal Components by Using LSTM Model

Through a large number of experiments and years of tests by Mr. Huang [24], it has been found that the eigenmode component of the pseudo-component or noise concentration is separated during the empirical mode decomposition process. It is an important issue about how to select effective components from multiple components in signal recovery [25]. 

Formula (8) shows that the intrinsic mode component of a signal can be obtained by empirical mode decomposition. Due to the decomposition error, the effective intrinsic mode component of B term and the pseudo component of C term or the concentrated component of noise can be generated.

(8) $$\sum_{i=1}^{a}c_{i}=\sum_{j=1}^{b}c_{j}+\sum_{l=1}^{c}c_{l}$$

The correlation between the intrinsic mode components and the pre-decomposed signals obtained by empirical mode decomposition is as follows:

(9) $$\begin{array}{ll} R_{h_{4}\left(t\right),c_{i}^{\prime }} & =E\left[h_{4}\left(t\right)*c_{i}^{\prime }\left(t+\tau \right)\right]=E[\sum_{j=1}^{a_{1}}c_{j}\left(t\right)*c_{i}^{\prime }\left(t+\tau \right)]\\ & =E\left(c_{1}\left(t\right)*c_{i}^{\prime }\left(t+\tau \right)\right)+\cdots +E\left(c_{a_{1}}\left(t\right)*c_{i}^{\prime }\left(t+\tau \right)\right)\\ & =R_{c_{i},c_{i}^{\prime }}\left(\tau \right)+\sum_{j=1,j\neq i}^{a_{1}}R_{c_{j},c_{i}^{\prime }}\left(\tau \right)\approx R_{c_{i},c_{i}^{\prime }}\left(\tau \right)\approx R_{c_{i},c_{i}^{\prime }}\left(\tau \right) \end{array}$$

Since the empirical mode decomposition process is a local orthogonal decomposition, it can be concluded from the premise:

(10) $$\sum_{j=1,j\neq i}^{a_{1}}R_{c_{i},c_{i}^{\prime }}\left(\tau \right)\approx 0$$

Then the above two formulas can be used to derive the correlation between the spurious component and the pre-decomposition signal. The above formula shows that the correlation between the decomposed intrinsic modal component and the original signal depends on the auto-correlation of each component’s autocorrelation. The correlation between the pseudo-component and the original signal is approximately zero. According to the non-directionality of random noise, the correlation between the components of the random noise and the original signal is low and approaches 0. Based on the above inference, we can make a provision. The correlation is judged *R* ≥ 0.02, and if it is greater than or equal to 0.02, it is recorded as an effective intrinsic modal component, and the self-adaptive selection is determined as the target of the next step by judging the correlation. However, through actual testing, it is found that the artificial correlation threshold will lead to incomplete classification and cannot be perfectly screened out all the effective intrinsic modal components. In order to screen out as many effective components as possible, we train an LSTM model here to continuously optimize the correlation threshold to enhance the classification effect [26].

In Figure 1, in order to filter out the effective natural mode components more effectively, the LSTM model is needed, Figure 2 describes the flow chart of RNN (recurrent neural network) model [27,28], compared with each other neutral network modules, RNN models have interconnected nodes among layers, which makes RNN perform well in dealing with timing problems. 

However, as the number of sequences in the RNN model increases, the amount of error loss in the feedback process will also continue to superimpose, which may cause the disappearance of gradients. In response to this problem, researchers proposed a more complex structural form, LSTM, as a hidden unit of RNN. Using LSTM model also improves the accuracy to a certain extent. The memory unit of LSTM is shown in Figure 3; and the flow chart of LSTM training is shown in Figure 4.

When we use serial index number I, *x* (*t*) represents the input of the inherent modal component. Similarly, *x* (*t* − 1) and *x* (*t* + 1) is the input of the inherent modal components when the serial index numbers *t* − 1 and *t* + 1 are used.

In this model, we use W matrices to represent the linear relationship parameters, which are suitable for the whole model.

In the hidden unit of the module, *x* (*t*) and *h* (*t* − 1) are used to determine the state of the forget gate f (*t*) that represents what information we’re going to throw (t indicates the serial number):

(11) $$f(t)=\mathrm{sigm}\{W_{f}\cdot [h(t-1),g(x_{t})]+n_{f}\}$$

Where sigm() is a activation function, as shown in Formula (12), *n* is a bias of linear relation, and *g* (*x*) is a function for calculating the correlation of inherent modal components [29].

(12) $$\mathrm{sigm}(x)=\frac{1}{1+e^{-x}}$$

And the input gate can calculates the cell state to be input, ${\tilde{C}}_{t}$ and the vector $i_{t}$ based on *x* (*t*) and *h* (*t* − 1) in Formulas (13) and (14) (*t* indicates the serial number):

(13) $${\tilde{C}}_{t}=\tanh\{W_{c}\cdot [h(t-1),g(x_{t})]+n_{c}\}$$

(14) $$i_{t}=\mathrm{sigm}\{W_{i}\cdot [h(t-1),g(x_{t})]+n_{i}\}$$

Where tanh() is a activation function, as shown in Formula (15):

(15) $$\tanh(x)=\frac{e^{x}-e^{-x}}{e^{x}+e^{-x}}$$

And the old cell state $C_{t-1}$ can be updated by calculating with the results of the forget gate and the input gate in Formula (16):

(16) $$C_{t}=C_{t-1}*f_{t}+{\tilde{C}}_{t}*i_{t}$$

Output gate calculates the output gate state, *o*(*t*), and the cell state $C_{t}$ determines what information in *o*(*t*) will be output units.

(17) $$o(t)=\mathrm{sigm}\{W_{o}\cdot [h(t-1),g(x_{t})]+n_{o}\}$$

(18) $$h(t)=o_{t}*\tanh(C_{t})$$

At the end of the series index number t, our predicted output is as follow:

(19) y^(t)=sigm[Wy⋅h(t)+ny]

Finally, we used the log likelihood function *L* (*t*) to quantify the loss of the model at the current position, compare the differences between *y* ^ (*t*) and *y* (*t*) [30].

### 2.4. Reconstructing and Enhancing Weak Signals 

The intrinsic modal component is a stationary signal or a simple non-linear signal and belongs to a narrowband signal. Any narrowband signal *X*(*t*) can get its Hilbert transform result *Y*(*t*). The formula is as follows:

(20) $$Y\left(t\right)=\frac{1}{\pi }\int_{-\infty }^{\infty }\frac{X\left(\tau \right)}{t-\tau }d\tau$$

For the selected effective modal components, the Hilbert transform is used to construct the analytical signal:

(21) $$Z_{k}\left(t\right)=X_{k}\left(t\right)+iY_{k}\left(t\right)=a_{k}\left(t\right)e^{i\theta_{k}\left(t\right)}$$

(22) $$a_{k}(t)=\sqrt{X_{k}^{2}(t)+Y_{k}^{2}(t)}$$

(23) $$\theta_{k}(t)=\arctan\frac{Y_{k}(t)}{X_{k}(t)}$$

(24) $$a_{k}(t)=\sqrt{X_{k}^{2}(t)+Y_{k}^{2}(t)}$$

Instantaneous phase and amplitude can be used to recover weak signals:

(25) x~(t)=Re∑k=1na~k(t)eiθk(t)

Traditional signal enhancement methods are very sensitive to noise, which can cause significant overshoots that can cause signal blurring. Here we use artificial training GAN (generative adversarial network) to generate high-resolution signals.

In order to improve the stability and efficiency of training, we adopt an incremental enlargement method to train GAN, as shown in Figure 5:

When the real seismic signal data input into the discriminator, we must make the objective function to be maximized as much as possible thus that the machine can determine that it is the real data. The second half of the formula shows that the generator makes the function *G* (*z*) as small as possible when inputting and generating real seismic data. In this process, the generator deceives the discriminator, making it mistakenly believe that the input is factual data [31], and the discriminator tries to identify it as fake data. They train with each other to reach the Nash equilibrium.

We start training with generators (*g*) and discriminators (*d*) with low spatial resolution, with a resolution of 4 × 4 at the beginning, and then add a convolution layer to G and D after each training, thus as to gradually improve the spatial resolution of the generated signal [32,33,34,35]. All involved convolution layers can be retrained in the whole training process. N × N in the figure refers to the convolution layer working at N*N spatial resolution. 

We give the distribution of reconstructed signal data Pdata (x), and distribution of Pg (x, θ), which is controlled by θ. The formula can be found in Appendix A.

We complete GAN training based on KL divergence [36] and get the final signal enhancement model, the reconstructed signal can be steadily enhanced by adding layers from low to high.

## 3. Experimental Results and Discussion

This section will be divided into two parts. First, we will introduce the model training and parameter setting in the experimental process, and then we will compare and analyze different signal processing methods. The framework of this section is shown in Figure 6.

### 3.1. Training Detail

The LSTM model used in this paper contains two LSTM layers, a dropout layer with *p* = 0.2, a fully connected and a sigmoid layer. The LSTM gets 32 hidden units and the loss function is the log likelihood function. We also used the Adam optimizer to train the network. The learning rate was 0.01, which was attenuated by the natural index, the batch size was 20, and the number of the epoch was 500. The change of loss value of the model is shown in Figure 7. When the model was trained 400 times, it basically converged, and the final loss value was around 0.015. 

When training GAN, the reconstructed weak signal was used as input. In the generator, we used relu as the activation and tanh as the activation function in the last layer. In the discriminator, we used leakyrelu as the activation function. In one epoch, we trained the discriminator at first. After an epoch, we froze the weight of the discriminator and trained the generator. At the end of each epoch, we added a 2 × 2 convolution layer to the generator and discriminator. During model training, we set a batch size of 16, and we iterated 300 epochs. We used an Adam optimizer, and the initial learning rate was set to 2 × 10^−4^, which was reduced to 2 × 10^−5^ after 40 rounds of training.

### 3.2. Contrast and Verification

In the field of biomedicine, mechanical failure, and geophysics [37], the status of weak signals is prevalent. In order to verify the validity of the method, we chose the 3D weak seismic data in the field of geophysics as the test target for experimental testing. 

In seismic exploration, people used artificial methods to cause crustal vibration (such as explosive explosion and vibriosis vibration), then they used precision instruments to record the vibration information of each receiving point on the ground after explode, and people finally inferred the underground geological structure according to the result that processed from the original record information. When seismic waves travel underground, it will encounter different rock stratum interfaces with different media, which will produce reflection and refraction. At this time, we can receive this kind of seismic wave with geophone on the surface. The seismic signals we receive are related to the characteristics of seismic source, the location of the detection point, and the nature and structure of the underground strata where the seismic waves pass. Through the processing and interpretation of seismic wave records, we can infer the nature and shape of underground rock strata. The acquisition of the seismic signal is shown in Figure 8.

When effective waves are generated, various interference waves will also be generated. According to its generating law, it can be divided into regular noise and random noise. Regular noise has a dominant frequency and apparent velocity, its apparent velocity, apparent frequency, and waveform all have their own propagation characteristics and rules. It can be suppressed according to differences in the frequency spectrum or propagation direction between it and the effective wave. Random noise is the interference wave without a certain frequency and apparent velocity, which is mainly generated by natural and human factors. The method proposed in this paper is mainly to suppress this kind of random noise, highlight the effective signal, and achieve signal enhancement.

#### 3.2.1. Experimental Results and Analysis of Synthetic Weak Signal Data

In order to detect the efficiency of our approach, we tested some simulated 3D seismic data. In our synthetic 3D seismic data, in the horizontal direction, each dataset has 50 seismic traces, each trace has 500 seismic sampling points, the plane in the horizontal direction is shown in Figure 9. We use the *x*-axis to represent the amount of analog 3D seismic data channels, and the *y*-axis is the vertical sampling points of analog 3D seismic data. Figure 9a shows the profile formed by the first line, which consists of a horizontal and a slanting reflection axis. Figure 9b is the profile of the first line after convolution of the reflection axis and the Ricker wavelet in the whole data. Figure 9c is a profile of the first line after Gaussian white noise is added to the whole synthetic data volume. Figure 9d is a profile of the first sideline of the synthesized 3D data processed by our method. 

To test the feasibility of our method, we also did the contrast experiments of different methods in the background with strong noise. Figure 10a is a section diagram with Gaussian white noise and a signal-to-noise ratio of 0.5. Figure 10b shows a section diagram enhanced by wavelet transform. Figure 10c shows a section diagram enhanced by a curved wave transform. Figure 10d shows a section diagram enhanced by our method.

Figure 11 shows that the profile of the sideline was composed of two reflection axes in the same direction at the beginning. After being convoluted with the wavelet, some parts of the two reflection axes in the same direction were indistinguishable. After being processed by our method, two coaxial axes can be distinguished clearly. In order to reflect the results of different methods more intuitively, we used Formula (22) to calculate the SNR of 10 lines of the composite data and the SNR before processing, *g* (*x*, *y*) was the original 3D seismic data and *g* ^ (*x*, *y*) represented the denoised 3D data. A is the number of seismic trace and B is the number of vertical sampling points. The formula is shown in (26):

(26) $$\begin{array}{l} \mathrm{SNR}=20\log_{10}\frac{\sum {}_{x=0}^{A-1}\sum {}_{y=0}^{B-1}{\left[\hat{g}(x,y)\right]}^{2}}{\sum {}_{x=0}^{A-1}\sum {}_{y=0}^{B-1}{\left[g(x,y)-\hat{g}(x,y)\right]}^{2}} \end{array}$$

The comparison results are shown in Figure 11. In Figure 11, the *y*-axis represents the SNR, and the *x*-axis represents the 10 data lines processed by the composite data. The result shows that the SNR of EMDNN processed is higher than others in the background of strong noise. The simulation results show that the 3D data processed by this method can clearly identify the wedge-shaped geology, which shows that EMDNN method not only improves the SNR but also increases the resolution.

#### 3.2.2. Experiment and Analysis of Actual Weak Signal Data

Next, we conducted experiments on the actual weak reflection 3D data. The actual three-dimensional seismic data that we took were the weak seismic signal hidden in the background of strong noise. There were 1160 lines in the data, 1040 for each line, 6000 ms for each seismic signal and 1ms for sampling interval. We processed the whole three-dimensional seismic data, and then observed the profile of a survey line, and took the profile with weak reflection seismic signal, which contained 100 channels of 600 sampling points. The effect comparison before and after processing is shown in Figure 12 (the red rectangle represents the most distinct area before and after processing). Figure 12a is the unprocessed figure of the profile of the sideline, and Figure 12b is the figure that has been recovered by the wavelet transform. Figure 12c is a graph that has been recovered by curved wave transformation. Figure 12d is the graph that has been recovered by this method. Figure 12 shows that the pre-processing signal cannot be recognized at all. After wavelet and curve transform processing, compared with the original signal, some weak signals were recovered obviously, but some of the same direction axes were still difficult to distinguish. As a result, the effect of the data processed by our method was obviously improved, and the weak signal was clearly reflected. Figure 13a,c were unprocessed figures of the sections of different sidings, and Figure 13b,d were the figures intercepted after the processing by our method. It shows that the geological horizon processed by our method was clearer.

#### 3.2.3. Parallel Processing Experiments and Analysis

In order to verify the advantage of this method in processing speed, we selected five groups of actual seismic weak signal data of different sizes as experimental objects, and used non-parallelized algorithms (CPU processing) and parallelized algorithms (GPU processing) to process the experimental data [38]. We counted and tabulated the processing time of the two methods. The results are shown in the Table 1. The experimental results in Table 1 show that the processing time of the GPU parallelized algorithm was only one-fifth of the conventional CPU processing time, which improves the efficiency of processing.

According to the comparison experiment, we know that using the GPU’s powerful parallel processing capability can effectively improve the program’s operating speed and reduce the processing and reconstruction time of weak signals. When the processed data was small, the acceleration ratio was only 2–4 times because all the thread resources on the GPU cannot be fully utilized. As the amount of processing data increased, all thread resources on the GPU were mobilized, and the speedup ratio gradually increased. When the amount of data processed exceeded 10 G, the processing speed was increased by nearly 8 times. The processing time and reconstruction time of the massive weak signal data were greatly reduced, the working time of the processing personnel was saved, and the working efficiency was improved.

## 4. Conclusions and Future Work

This paper proposes a weak signal enhancement method based on the EMDNN model for the characteristics of weak signals. Through theoretical and experimental results, it is shown that the weak signal of the typical field is selected for processing experiments, and the signal-to-noise ratio of the recovered weak signal is significantly improved. This method uses GPU parallel computing to solve the shortcomings of the large amount of computation and slow operation speed, which is 4–5 times faster than conventional CPU. After trying to introduce the LSTM model and GAN model into traditional weak signal reconstruction and enhancement methods, we find that further breakthroughs have been made in adaptive and weak signal image enhancement, which greatly improves the signal-to-noise ratio. With the development of research, we will study the application of gated recurrent unit (GRU) model in selecting the natural mode components in empirical mode decomposition and study the varieties of the generative adversarial network to improve the effect of signal enhancement further.

## Figures and Tables

**Figure 1:** Flow chart of the weak signal reconstruction method under the neural network-assisted empirical mode decomposition (EMDNN) model.

**Figure 2:** The flow chart of the recurrent neural network (RNN) model.

**Figure 3:** Long short term memory (LSTM) internal unit structure diagram.

**Figure 4:** The flow chart of LSTM training.

**Figure 5:** The flow chart of generative adversarial networks (GAN) enhancement.

**Figure 6:** The flow chart of the experimental process.

**Figure 7:** The chart of training process of LSTM model.

**Figure 8:** Flow chart of seismic signal acquisition.

**Figure 9:** The chart of processed synthetic seismic data; (**a**) the profile of reflection coefficient; (**b**) the convoluted profile; (**c**) the profile after adding noise; (**d**) the processed profile by EMDNN method.

**Figure 10:** The chart of Wedge model between the original and processed: (**a**) The wedge model under strong noise background; (**b**) processed wedge model using the wavelet transform; (**c**) processed wedge model using the curvelet transform; (**d**) processed wedge model using EMDNN method.

**Figure 11:** The contrast chart of SNR (original and the processed simulated data).

**Figure 12:** The comparison among different processing method; (**a**) original seismic data; (**b**) the seismic data processed by the wavelet transform; (**c**) the seismic data processed by the curvelet transform; (**d**) the seismic data processed by our method.

**Figure 13:** Actual seismic data processing; (**a**) actual seismic profile; (**b**) profile 1 processed by this method; (**c**) actual seismic profile; (**d**) profile 2 processed by this method.

**Table 1:** The comparison of processing speed between CPU and GPU.

Test Data	Data Size (mb)	CPU Program Running Time (s)	GPU Program Running Time (s)	Speed up Ratio
Data1	43.2	32.03	12.41	2.58
Data2	262.8	256.15	68.49	3.74
Data3	568.7	532.47	122.69	4.34
Data4	1020.3	2209.41	355.78	6.21
Data5	14,328.8	40,160.92	5001.25	8.03

## Appendix A. KL Divergence Formula

$$\begin{array}{l} \theta^{*}=\arg\underset{\theta }{\max}\prod_{i=1}^{m}P_{G}(x^{i};\theta )=\arg\underset{\theta }{\max}\log\prod_{i=1}^{m}P_{G}(x^{i};\theta )\\ =\arg\underset{\theta }{\max}\sum_{i=1}^{m}P_{G}(x^{i};\theta )\\ \approx \arg\underset{\theta }{\max}Ex\sim Pdata[\log Pa(x;\theta )]\\ =\arg\underset{\theta }{\max}[\int_{x}Pdata(x)\log Pa(x;\theta )dx-\int_{x}Pdata(x)\log Pdata(x)dx]\\ =\arg\underset{\theta }{\max}\int_{x}Pdata(x)\frac{\log P_{G}(x;\theta )}{\log Pdata(x)}dx\\ =\arg\underset{\theta }{\min}\int_{x}Pdata(x)\frac{\log P_{G}(x;\theta )}{\log Pdata(x)}dx\\ =KL\\ G^{*}=\underset{\theta }{\min}\underset{\theta }{\max}V(G,D)\\ V=Ex\sim Pdata[\log D(x)]+Ex\sim Pa[1-\log D(x)]\\ =\int_{x}Pdata(x)\log D(x)\log D(x)+Pa(x)\log(1-D(x))dx\\ D^{*}=Pdata(x)\log D(x)+P_{G}(x)\log(1-D(x))\\ f(D)=a\log D+b\log(1-D)\\ \frac{df(D)}{dD}=a*\frac{1}{D}+b*\frac{1}{1-D}*(-1)=0\\ a*\frac{1}{D^{*}}=b*\frac{1}{1-D^{*}}\\ D^{*}=\frac{a}{a+b}\\ D^{*}(x)=\frac{Pdata(x)}{Pdata(x)+Pa(x)}\\ \max V(G,D)=V(G,D^{*})\\ =Ex\sim Pdata[\log\frac{Pdata(x)}{Pdata(x)+P_{G}(x)}]+Ex-Pa[1-\log\frac{Pdata(x)}{Pdata(x)+P_{G}(x)}]\\ =\int_{x}Pdata(x)\log\frac{Pdata(x)}{Pdata(x)+P_{G}(x)}dx+\int_{x}Pa(x)\log\frac{Pdata(x)}{Pdata(x)+P_{G}(x)}dx\\ JSD(P1∥P2)=1/2KL(P1∥\frac{P1+P2}{2})+1/2KL(P2∥\frac{P1+P2}{2})\\ \int_{x}Pdata(x)\log\frac{1/2*Pdata(x)}{\frac{Pdata(x)+P_{G}(x)dx}{2}}+\int_{x}P_{G}(x)\log\frac{1/2*Pdata(x)}{\frac{Pdata(x)+P_{G}(x)dx}{2}}\\ =2\log(1/2)+KL(Pdata(x)∥\frac{Pdata(x)+Pa(x)}{2})+KL(P_{G}(x)∥\frac{Pdata(x)+Pa(x)}{2})\\ =2\log(1/2)+2JSD(Pdata(x)∥P_{G}(x))\\ \to \underset{D}{\max}V(G,D) \end{array}$$
